# Research on Microseismic Source Location Method Based on Waveform Characteristics Monitored by Nanomaterial Sensor under the Background of Metal Oxide Polluted Environment

**DOI:** 10.1155/2022/5479007

**Published:** 2022-09-24

**Authors:** Shuai Wang, Zhaoxin Hu, Shasha Lu

**Affiliations:** ^1^School of Civil Engineering, Liaoning Technical University, Fuxin, Liaoning 123000, China; ^2^College of Mining, Liaoning Technical University, Fuxin 123000, China

## Abstract

In recent years, the monitoring range of source location technology has developed from being one-dimensional and two-dimensional to being three-dimensional. However, due to the complexity and nonuniformity of the seismic wave propagation medium and the uncertainty of the propagation law, there will be large errors in the source location results. Therefore, the analysis of vibration signal has become the key problem of current research. This paper designs a microseismic monitoring system based on Internet of Things sensors, which can monitor the vibration wave characteristics of vibration signals. In order to test the positioning accuracy of the system, this paper introduces three positioning methods: target positioning method based on time difference, time delay estimation method based on EMD, and source target positioning method based on the characteristic frequency of vibration signal. The purpose of this paper is to find the most accurate method from the three source location methods. Through these three methods, the vibration source generated by a single person walking in situ can be located in the vibration positioning experiment of human walking. The error between the actual position and the measurement source position is compared. The results show that the time delay estimation method based on empirical mode decomposition has the highest positioning accuracy. In addition, in the microseismic experiment, it is proved that the positioning accuracy of EMD using L1 norm statistical criterion is higher than that using L2 norm statistical criterion.

## 1. Introduction

At present, the most used microseismic source location technology is passive detection technology based on vibration sensor, which has great application value in both military and civil aspects. However, the positioning accuracy of this technology is still a difficulty in unattended ground sensor technology. Therefore, it is very necessary to study a precise location technology of source location. Microseisms are broadly divided into engineering microseisms and naturally occurring microseisms. One of the most obvious features of the waveform is its short duration, which is generally only a few tenths of a second.

At present, many scholars have conducted in-depth research on the microseismic source location method based on the monitoring wave characteristics of IoT sensors and have achieved good results. For example, some developed countries have begun to study the application of ground motion sensors to detect ground targets in practice. Small amplitude is also an important criterion for distinguishing microseismic signals. Microseismic waves are not different from seismic waves in physical nature and can be understood as seismic waves with small energy. In the UGS system used by border defense, the acoustic shock sensor is mainly used to detect and identify ground intrusion targets. Some areas install UGS on highways, and vibration sensors can monitor ground vehicles at any time, or UGS systems are used for border protection and highways [1, 2]. Note that the core and foundation of the Internet of Things, which is an extended network based on the Internet, are still the Internet. In addition, its client extends to any goods for information exchange and communication. Some scholars have studied the human vehicle detection system based on vibration sensors, analyzed the principle of vibration detection, completed the design of the detection system through software and hardware research, and realized the detection and alarm functions [3]. Compared with traditional sensors, optical fiber sensors have many characteristics: high sensitivity, simple structure, small volume, corrosion resistance, good electrical insulation, flexible optical path, easy-to-realize telemetry, and so forth. The combination of optical fiber sensor and integrated optical path technology accelerates the development of optical fiber sensor technology. A researcher has studied the projectile landing point positioning technology based on the shock sensor and verified the effectiveness of the positioning algorithm by analyzing the vibration signal generated when the projectile landed [4]. Although there are many methods for locating microseismic sources, there is still a certain gap to achieve accurate positioning.

This paper introduces two microseismic monitoring technologies, acoustic wave detection technology and acoustic emission technology, and then proposes four hypocenter location methods. According to the application of three methods in the IoT sensor microseismic monitoring system, the source location simulation experiment is carried out. The results show that the EMD-based time delay estimation positioning method has more advantages than the other two positioning methods. Note that acoustic emission technology has become a powerful tool for experimental stress analysis, which can be used to detect cracks, study the corrosion fracture process, and monitor the fatigue fracture propagation of components. Acoustic emission technology can also be used to evaluate the integrity of components and judge the danger degree of structures.

The innovation of this paper is to measure the positioning accuracy of three positioning methods and conduct two experiments of human walking vibration source positioning and microseismic event vibration source positioning and introduce norm statistical criteria to compare positioning errors and event residuals.

## 2. Microseismic Source Location

### 2.1. Overview of Microseismic Monitoring Technology

Among the many technologies that use sound waves to study the properties of materials, they can be divided into sound wave detection technology and sound emission technology according to the source of sound waves. Acoustic detection technology typically uses two sensors with different functions. One of the sensors emits a wave signal, which is transmitted into the natural environment, and the signal is then received by the other sensor. Comparing the arrival time, phase, amplitude, and so forth of the transmitted wave signal with the parameters of the received wave signal, we can know the current environmental state [5]. Acoustic detection techniques include seismic exploration in nature, recording the depth of the crust, detecting ultrasonic flaws in samples in the laboratory, and measuring the velocity of elastic waves. The working principle of the acoustic emission instrument is that the sensor made of piezoelectric crystal is coupled to the test piece to be tested. After receiving the acoustic emission signal, it converts the weak mechanical vibration into an electrical signal, which is amplified by the preamplifier, and then the mechanical noise is removed by the filter, and then the signal is further amplified by the main amplifier for signal processing. Acoustic emission technology only uses the receiving sensor(s), which can understand the stress state and damage rupture process of the material based on the shock wave signal. Seismic monitoring, microseismic monitoring, rock explosion warning, and laboratory characterization of rock material damage and fracture acoustic emission all belong to the category of acoustic emission research [6].

Sonic detection technology detects defects such as cracks and material failures by comparing and analyzing transmitted and received sound waves. Acoustic emission technology analyzes the waveform, calculates the time and location of rupture, and receives the shock wave signal generated by the material in the process of damage or rupture. The advantages of acoustic detection are large thickness, high sensitivity, fast speed, low cost, and the ability to locate and quantify defects. Therefore, it can not only control the defects in the material but also infer the formation process and trend of the defects [7]. Because of the above characteristics and advantages of acoustic emission technology, it has been rapidly developed and widely used in geotechnical mechanics and engineering.

A large number of scientists at home and abroad have carried out very detailed research on the acoustic emission activity of metal materials. Plastic deformation of metallic materials is generally considered to be the main source of acoustic emissions. From a macroscopic point of view, crack propagation, fatigue damage, stress corrosion, and hydrogen embrittlement are the main sources of acoustic emission. Stress corrosion refers to the destruction of metal in corrosive medium under the action of tensile stress. This kind of corrosion generally passes through grains, which is called transgranular corrosion. Stress corrosion is the process of material failure caused by the combined action of strain and corrosion caused by residual or applied stress. The fracture of materials caused by stress corrosion is called stress corrosion fracture. From a microscopic point of view, the emission of acoustic signals is mainly related to displacement expansion [8]. The hardware and software systems for microseismic monitoring developed rapidly; in addition, acoustic emission/microseismic monitoring theory, experimental research, and field tests were carried out during this period, laying the foundation for the industrial application of microseismic monitoring. Bloem et al. analyzed the temporal and spatial distribution of more than 2,000 microseismic events and found that there is a direct connection between mining support and the distribution of microseismic events [9]. Dukanac studied the statistical relationship between microseismic activity and mineral recovery rate and used the seismic energy released during the period to evaluate the mine earthquake risk of coal mines.

### 2.2. The Method of Locating the Source Target

#### 2.2.1. Target Positioning Method Based on TDOA

The basic idea of the TDOA localization method is that the equation can be obtained by the difference between the distances between the target of the unknown source and the two sensors. When there are many sensors, many equations can be identified between the target and the unknown source sensor, and then the target position can be determined through the equation intersection, and the equation solutions that do not meet the requirements can be excluded, which is also a manifestation of the overcharacterization of the TDOA positioning method. However, the distance difference in the solution process must be known to obtain the target solution of the equation. Once the wave speed is known, calculating the time difference of arrival becomes a key problem in the positioning process. The TDOA localization method is used to estimate the position of the source target which first needs to calculate the time required to reach the two sensors of the target signal and then obtain the position of the source target [10].

#### 2.2.2. EMD-Based Time Delay Estimation and Positioning Method

Delay estimation is the key to TDOA positioning methods. Commonly used interconnect delay estimation methods are often used to analyze static signals with less noise, but real signals are often nonstationary noise signals. Given the sensitivity to noise, many scientists have improved it. The basic principle of EMD-based source location is to empirically decompose the original signal, and, according to the energy distribution of each signal reconstruction element, the IMF component that best matches the target characteristics is selected, which can be reduced. Empirical mode decomposition decomposes the signal according to the time scale characteristics of the data itself, without setting any basis function in advance. This is essentially different from Fourier decomposition and wavelet decomposition based on a priori harmonic basis function and wavelet basis function. Intervening on unnecessary parts and preserving key features of the signal improve the accuracy of latency estimation. Since the useful frequencies of the collected real signal are concentrated in the low frequency band, this method is similar to an adaptive low-pass filter [11].

#### 2.2.3. Seismic Target Location Method Based on Characteristic Frequency of Vibration Signal

The time-delay estimation and positioning method based on EMD has certain limitations. Because such methods have certain requirements on the signal-to-noise ratio of the signal, according to the instability and low frequency characteristics of the vibration signal, the local mean decomposition (LMD) is used to divide the signal into thousands of instantaneous frequencies to obtain the standard signal frequency, and the time delay is calculated according to the first appearance time of the characteristic frequency. Both LMD and EMD are adaptive decomposition methods based on the extremum point information of the signal itself, and the decomposition results are several component signals from high frequency to low frequency. The main difference is that the solution method is different and the decomposition result is different. The local mean decomposition can decompose the signal locally through the moving average, while the spline interpolation method is used in the EMD method. The local mean decomposition method adaptively decomposes a complex nonstationary multicomponent signal into the sum of several physically meaningful product functions of instantaneous frequencies, in which each component is directly obtained from an envelope signal and a pure FM signal. Further, by combining the instantaneous amplitude and instantaneous frequency of all PF components, the complete time-frequency distribution of the original signal can be obtained. The LMD process obtains the product function, and the EMD obtains the intrinsic mode function. Compared with the IMF component, the PF component contains more amplitude and frequency information, and its physical meaning is clearer [12]. Vouillamoz et al. took landslide clay debris on landslides caused by microseisms as research objects, and used the LMD method to collect the vibration frequency of clay after microseisms. Due to its high complexity, it is difficult to analyze microseismic signals of clay debris [13].

#### 2.2.4. Relative Positioning Method

The relative positioning method is a method of locating the seismic source by inputting the arrival time difference of the first detection base station. The basic principle of the relative positioning method is as follows: determine the initial time difference received from the sensor base station, combine the travel time equation between the source and the sensor, and establish the travel time equation between the source and the sensor through the arrival time difference of the first arrival wave received in the sensor base station and combined with the positioning algorithm to complete the location of the source. Hossein et al. used the relative positioning method to locate the microseismic events in the mining area, locate the source of the earthquake through the sensor base station in the mining area, and determine the cause and magnitude of the microseismic event in the mining area [14].

### 2.3. Covariance Matrix Method for Polarization Positioning

The basic idea of polarization analysis is to use the covariance matrix method to obtain the main polarization direction of the wave in a time window, and then, according to the polarization characteristics of the data, the projection formula is improved to separate the wave field. Then the covariance matrix method is used to solve the eigenvalues and eigenvectors of the covariance matrix and further obtain the azimuth angle and incidence angle of the source propagation direction. In the adaptive covariance matrix, set the three-component data *u*_*i*_(*t*) (*i* = *N*, *E*, *D*), find the Hilbert transform spectrum *u*_*j*_^*h*^(*t*) of the three-component data, and obtain its analytical signal:

(1) $$\begin{array}{c} C_{i}\left(t\right)=u_{i}\left(t\right)+ju_{i}^{h}\left(t\right). \end{array}$$

The local signal around time *t* can be approximated using the analytical signal *C*_*i*_(*t*).

(2) $$\begin{array}{c} u_{i}\left(t+\tau \right)\approx \frac{1}{2}\left(C_{i}\left(t\right)e^{j\Omega_{i}\left(t\right)\tau }+C_{i}^{*}\left(t\right)e^{-j\Omega_{i}\left(t\right)\tau }\right). \end{array}$$

In the above formula, Ω_*I*_(*t*) represents the instantaneous frequency, and *τ* is a parameter.

## 3. IoT Sensor Microseismic Monitoring System Design

### 3.1. Establishment of Sensor Space Coordinates

At present, the influence of sensor spatial coordinates on the accuracy of source location is relatively small. Microseismic sensors are usually located in underground space or on the surface, and the accuracy of their spatial coordinates mainly depends on the sensitivity of the measuring instruments. In the early stage of establishing a microseismic monitoring system, it is necessary to measure the spatial coordinates of all sensors in the monitoring system and ensure that the spatial coordinates correspond to the microseismic sensors one by one. The multichannel microseismic monitoring system is used to monitor the stability and safety of underground engineering, which breaks through the traditional monitoring mode in the sense of “point” or “line” in force and displacement. It is the monitoring of the spatial and temporal process of rock failure process within the scope of excavation influence. This method is easy to realize the monitoring of places that are inaccessible to people in conventional methods. During the operation of the microseismic monitoring system, some sensors may need to be adjusted due to the change of the microseismic monitoring area. Therefore, it is necessary to record the detailed information of each sensor and create a microseismic sensor and adjust the information table to ensure that the sensor has been changed and the spatial coordinates are accurate.

Regularly (e.g., 3 months) spatially check the spatial coordinates of all sensors in the microseismic monitoring system. There is 24-hour continuous monitoring of all sensor-controlled vibration wave signals. If sensor inactivation, signal loss, or abnormal signal is found, corrective measures should be taken in time. Full digital technology overcomes the shortcomings of analog signal system, makes computer monitoring possible, and makes data acquisition, processing, and storage more convenient. Due to the large amount of data collected by the multichannel monitoring system, the computer is required to process the data in real time and save it. The large capacity hard disk storage devices, optical disks, and other media provide a guarantee for the storage, long-term storage, and reading of the recorded data.

### 3.2. Microseismic Network Layout

A large number of studies have shown that the advantages and disadvantages of the microseismic network layout plan are the key factors in determining the accuracy of the source location. However, the mechanism of the microseismic network on the source location has not received enough attention and in-depth systematic research. At present, the network layout focuses on optimizing the design of the network, while the internal relationship between the microseismic network and the source location and the mechanism of the network on the source location are less studied and have not been fundamentally resolved. With the continuous improvement of the requirements for the accuracy of the source location, the influence mechanism of the microseismic network on the source location accuracy and the optimal arrangement of the microseismic network will become the focus of future research on the microseismic location monitoring. Generally speaking, the influence of microseismic network on source location is mainly reflected in the two following aspects: one is the number of sensors in the network, which is called the scale of the microseismic network; the other is the influence of the spatial layout of the microseismic network on the location of the source mechanism.

### 3.3. Design of Epicenter Location System Based on IoT Sensors

The Internet of Things is another area of the Internet that deserves attention after the standards-based Internet has self-discipline management capabilities. Network nodes in IoT are objects that have their own identities and actively participate in information exchange. Analyzing the specific definition, the Internet of Things covers wireless sensor networks. Cloud computing aims to integrate multiple relatively low-cost computing entities into a perfect system with strong computing power through the network and enable end users to get these powerful computing services with the help of advanced business models. A core idea of cloud computing is to continuously improve the processing capacity of the “cloud,” continuously reduce the processing burden of user terminals, and finally simplify it into a simple input and output device. Whether it is reconnaissance or surveillance network, wireless sensor network only supports the exchange of information between objects; the purpose is to provide users with the information required by the environment. Therefore, the wireless sensor network is the technical basis of the Internet of Things and a branch network of the Internet of Things.

The architecture of the entire source location system based on IoT sensors is shown in Figure 1. The source location system based on IoT sensors is composed of wireless sensors, multichannel switch boxes, data acquisition instruments, and host computers. The sensor nodes collect environmental data and transmit them to the gateway through radio frequency. The gateway transmits the data to the host computer through wired or wireless media. Sensor nodes work periodically to collect environmental data. Wireless sensor network is a kind of sensor network composed of independent distributed nodes and gateways. Sensor nodes placed in different locations constantly collect physical information of the outside world, such as temperature, sound, and vibration. Independent nodes communicate with each other through wireless networks. Each node of wireless sensor network can realize the collection and simple data processing and also receive data from other nodes and finally send the data to the gateway. By artificially changing the state of the node, the working and dormant states of the node are replaced, and the gateway node coordinates the entire wireless sensor network. The gateway periodically sends time synchronization messages to the network to keep all sensor nodes synchronized over time and then completes the monitoring and transmission of environmental information together. In addition, the gateway is also responsible for receiving the command sent by the above computer and transmitting it to the sensor node, and the sensor node is responsible for receiving and executing the command.

## 4. Microseismic Monitoring System Positioning Simulation Experiment

### 4.1. Standing Still

#### 4.1.1. Comparison of TDOA-Based and EMD-Based Positioning Methods

In the test, people walked in place at 1, 3, 6, 9, and 12 meters away from the IoT sensor, while the sensor distances were 1, 3, and 5 meters, respectively. The signal was the vibration generated by a single person walking in place. In this paper, the collected position calculation measurements of the source and target positions are compared with the initial settings between the person and the sensor, and the results are shown in Tables 1–3. The footstep signal 12 meters away from the center of the sensor layout is weak. The method cannot obtain the estimated time delay, so only the positioning measurements of 1 m, 3 m, 6 m, and 9 m are obtained. The data units in the table are all m.

When the IoT sensor distances are 1 m, 3 m, and 5 m, the positioning accuracy of the TDOA-based positioning method is 86.35%, 88.28%, and 86.94%, respectively, and the positioning accuracy of the EMD-based positioning method is 91.44%, 93.65%, and 92.07%, no matter how far the sensor distance is and how far the stepping signal is between the person and the sensor, the time delay estimation accuracy based on EMD method is higher than that based on TDOA positioning method, and the error is small. Moreover, it can also be found that the sensor distance has a certain influence on the positioning results. When the sensor distance is 3 meters, the positioning error is smaller than that when the sensor distance is 1 meter and 6 meters, which will affect the positioning accuracy. It should take a lot of experimentation to find the most suitable spacing.

#### 4.1.2. The Source Location Results Based on the Target Eigenfrequencies

In the experiment, multiple collections were carried out under different IoT sensor distances, and people stepped on the spot at 1, 3, 6, 9, and 12 meters away from the center of the equilateral triangle of the sensor. Perform positioning analysis on the collected signals at different distances. The positioning results are shown in Table 4, and Figure 1 shows the positioning error based on the target adjustment frequency.

From the error results in Figure 2, it can be seen that the positioning error when the sensor distance is 3 m is smaller than that when the distance is 1 m and 5 m, indicating that the closer the sensor is, the more accurate the positioning is. When the distance is too close, the collected seismic waves will contain other waves than thunder waves, resulting in larger positioning errors. When the water wave meets the interface, it will be reflected back from the boundary, forming a series of water waves transmitted to the outside of the bank, which overlap with the water waves transmitted to the inside of the bank. When the ocean wave slants into the shoal, the wave moves slowly when the depth of the sea becomes shallow and falls behind the wave in the deeper water. The result is that the wave bends towards shallow water.

#### 4.1.3. Comparison of Positioning Accuracy of Three Positioning Methods

Figure 3 shows the comparison of the positioning method based on TDOA, the positioning accuracy based on the characteristic frequency of the ground motion signal, and the positioning accuracy based on the EMD delay estimation. Combining Table 4 and Figure 1, it can be seen that regardless of the distance between the IoT sensors, the positioning accuracy of the method based on the characteristic frequency of the ground motion signal is higher than that of the EMD-based time delay estimation method and the TDOA-based positioning method. When the noise is large, the phenomenon of not getting the delay estimation value will not occur. The EMD delay estimation positioning method and the TDOA-based positioning method cannot be used. Target positioning is at a distance of 12 meters.

In summary, when the propagation distance of the shock wave is large, its energy is continuously attenuated during the propagation process, and the signal-to-noise ratio is reduced. The positioning result has a large error. When the seismic wave propagation distance is small, the existence of various waves and environmental noise and other factors will also lead to increased errors. Therefore, the distance between IoT sensors must be suitable to minimize the positioning error and maximize the positioning accuracy.

### 4.2. Microseismic Location

The hypocenter location error refers to the difference between the calculated hypocenter and the real hypocenter, but, in practical applications, the actual location of the microseismic event is unknown. In order to further verify the superiority of the positioning method based on EMD delay estimation, the L1 norm statistical criterion and the L2 norm statistical criterion were used to locate eight microseismic events, and the positioning errors and event residuals were compared. The results are shown in Figure 4. According to the point source model, only two nodal planes of the earthquake can be determined according to the far-field P-wave and S-wave observations, and it is impossible to determine which of them is the actual fault plane. In order to identify which is fault plane, it is necessary to supplement other information about the source, such as surface rupture data, spatial distribution characteristics of aftershocks, and shape of isoseismal lines in the polar region.

It can be seen from Figure 4 that, for the positioning method based on EMD delay estimation, there is an obvious positive correlation between the event residual and the source positioning error. Generally, the larger the event residual, the greater the positioning error; and, based on the L1 norm statistics, there is no positive correlation between the event residuals obtained by the source location method based on the criterion and the L2 norm statistical criterion and the source location error. For example, when the L1 norm statistical criterion is used, the event residuals of the third and sixth microseismic events are both 13.5 *μ*s, and the event residuals of the eighth microseismic test are 13.9 *μ*s, which are almost the same. However, their source location results are completely different. Their location errors are 16.4 m, 17.2 mm, and 18.4 mm, respectively. The L1 norm statistical criterion is obviously better than the L2 norm statistical criterion. In addition, the source location results show that, under the same input error, the location results using the L1 norm statistical criterion are generally better than the L2 norm statistical criterion, especially when there are outliers with large individual errors in the input data. The positioning accuracy of the L1 norm statistical criterion is much higher than that of the L2 norm statistical criterion. Besides, the basic idea of EMD method is to decompose the signal into a group of single component signal IMF combinations and then Hilbert transform each component to obtain instantaneous eigenvalues and transform these instantaneous eigenvalues to the first frequency plane to form Hilbert spectrum. In fact, EMD method is equivalent to defining a set of generalized bases with adaptive decomposition characteristics. From the perspective of traditional basis function definition, the adaptive generalized basis defined by EMD is an innovation of basis function in the field of signal processing.

## 5. Conclusion

Combining with the technology theory of the Internet of Things and introducing the concept of sensor network, a microseismic source monitoring system based on the Internet of Things sensors is designed, and the system is applied to the earthquake source location experiment. The positioning accuracy of three source positioning methods is compared in the human standing experiment, and it is concluded that the positioning method based on EMD delay estimation can be introduced into the source monitoring system to achieve precise positioning. In the microseismic location experiment, the location accuracy of the EMD location method based on the L1 norm statistic criterion is higher than that based on the L2 norm statistic criterion [15].

## Figures and Tables

**Figure 1:** Hypocenter location system architecture for IoT sensors.

**Figure 2:** Localization error based on target eigenfrequency.

**Figure 3:** Positioning accuracy comparison results.

**Figure 4:** Comparison of localization errors and event residuals.

**Table 1:** Target localization results when the sensor distance is 1 m.

	TDOA-based positioning method				EMD-based delay estimation			
Settings	1	3	6	9	1	3	6	9
Measurements	1.43	3.35	6.57	9.82	1.38	3.27	6.46	9.71
Error	0.43	0.35	0.57	0.82	0.38	0.27	0.46	0.71
Positioning accuracy	86.35%				91.44%			

**Table 2:** Target localization results when the sensor distance is 3 m.

	TDOA-based positioning method				EMD-based delay estimation			
Settings	1	3	6	9	1	3	6	9
Measurements	1.39	3.31	6.48	9.76	1.35	3.20	6.41	9.65
Error	0.39	0.31	0.48	0.76	0.35	0.20	0.41	0.65
Positioning accuracy	88.28%				93.65%			

**Table 3:** Target localization results when the sensor distance is 5 m.

	TDOA-based positioning method				EMD-based delay estimation			
Settings	1	3	6	9	1	3	6	9
Measurements	1.42	3.33	6.54	9.78	1.37	3.24	6.43	9.68
Error	0.42	0.33	0.54	0.78	0.37	0.24	0.43	0.68
Positioning accuracy	86.94%				92.07%			

**Table 4:** Source location results based on target eigenfrequencies.

	Settings	1	3	6	9	12
*L* = 1 m	Measurements	1.41	3.30	6.52	9.76	13.16
	Error	0.41	0.30	0.52	0.76	1.16

*L* = 3 m	Measurements	1.38	3.25	6.46	9.71	12.88
	Error	0.38	0.25	0.46	0.71	0.88

*L* = 5 m	Measurements	1.40	3.28	6.48	9.73	12.94
	Error	0.40	0.28	0.48	0.73	0.94

## Data Availability

The data underlying the results presented in the study are included within the manuscript.
